# Review of the Research Progress of Human Brain Oxygen Extraction Fraction by Magnetic Resonance Imaging

**DOI:** 10.1155/2022/4554271

**Published:** 2022-10-18

**Authors:** Zini Jian, Xianpei Wang, Meng Tian, Yufei Liu, Hongtai Yao, Li Gong, Bowen Li

**Affiliations:** ^1^School of Electronic and Electrical Engineering, Wuhan Textile University, Wuhan 430200, China; ^2^Electronic Information School, Wuhan University, Wuhan 430072, China; ^3^Hebei Xiong'an Taixin Technology Co., Ltd., Baoding 071000, China

## Abstract

In recent years, the incidence of cerebrovascular diseases (CVD) is increasing, which seriously endangers human health. The study on hemodynamics of cerebrovascular disease can help us to understand, prevent, and treat the disease. As one of the important parameters of human cerebral hemodynamics and tissue metabolism, OEF (oxygen extraction fraction) is of great value in central nervous system diseases. The use of BOLD (blood oxygen level dependent) effect offers the possibility to study cerebral hemodynamic and metabolic characteristics by MRI (magnetic resonance imaging) measurements. Therefore, this paper reviews the hemodynamic parameters of brain tissue, discusses the principles and methods of quantitative BOLD-based MRI measurements of OEF, and discusses the advantages and disadvantages of each method.

## 1. Introduction

Quantitative evaluation of brain tissue hemodynamics and metabolism, especially the relationship between brain function and oxygen utilization, is an important indicator for understanding normal brain function. The CMRO_2_ (cerebral metabolic rate of oxygen) refers to the oxygen metabolism of brain tissue and reflects the absolute value of the oxygen consumption of brain tissue [1]. OEF (oxygen extraction fraction) is defined as the ratio of blood oxygen that a tissue takes from the blood flow to maintain function and morphological integrity, and it reflects the efficiency of oxygen utilization by the tissue [2]. OEF and CMRO_2_ are the important markers of brain tissue activity and function [3, 4]. These quantitative evaluations have been used to study the pathophysiology of diseases such as brain tumors [5–7], stroke [8–10], Alzheimer's disease [11–13], Huntington's disease [14], Parkinson's disease [15], and other neurological disorders [16–19]. Raichle et al. and Gusnard et al. [20, 21] used OEF to determine the baseline status of normal human brains. When healthy human subjects are resting quietly with their eyes closed, although there are significant regional differences in cerebral blood flow and cerebral oxygen consumption metabolic rate [20, 21], the OEF diagram shows significant consistency, so that OEF can be used as a primary parameter of brain function [20–22]. The baseline state usually achieved when subjects are resting quietly but awake with their eyes closed can be described as the default mode of brain activity [23]. There was no significant difference in OEF values between gray matter and white matter of the brain and little variability in the population. So, OEF is suitable as a measurement index. Therefore, quantitative assessment of human brain OEF is very necessary for in-depth understanding of the pathophysiological status of a variety of diseases and subsequent treatment.

Currently, the clinically accepted gold standard for quantitative measurement of OEF is PET (positron emission tomography), which measures OEF by injecting ^15^O into the cervical vessels to obtain the difference of oxygen between arteries and veins [24–28]. However, the implementation of the PET method has many limitations. First of all, PET technology requires the production of radioisotope ^15^O by the accelerator as a tracer. ^15^O is not easy to prepare and obtain, and its half-life is very short. It can only be realized in the laboratory and cannot be carried out on a large scale in clinical practice [29]. Secondly, the spatial resolution of PET images is low. Last but not least, the implementation of PET technology requires exposure to ionizing radiation, which is harmful to human body [30]. These reasons have prevented PET technology from being widely used in human research and clinical practice.

With the rapid development of MRI (magnetic resonance imaging) technology, more and more studies have begun to study and process the blood perfusion and metabolism of brain tissue. MR (magnetic resonance) has the highest spatial resolution for brain lesions, and MRI is a safer and more comprehensive method in tissue structure, physiology, function, metabolism, and other aspects, especially in the diagnosis of nervous system diseases. Therefore, MRI has been gradually used in the diagnosis and prognostic treatment tracking of cerebrovascular diseases (CVD) such as stroke, and it has become a very important imaging tool. Compared with the previous OEF measurement methods, MRI measurement can be real-time, in vivo, and dynamic monitoring, and there is no ionizing radiation. It can accurately measure and calculate *R*2′ and finally fit the physiological parameters vCBV (venous cerebral blood volume) and OEF. The measurement of OEF value by MRI sequence can evaluate the physiological state of brain tissue disease in acute and chronic cerebrovascular diseases, which is of great significance for the clinical diagnosis and prevention of common cerebrovascular diseases. Therefore, if we can use MRI technology to measure OEF, it will undoubtedly promote its scientific research and clinical application. In this paper, we will focus on MRI-based OEF measurement methods and will discuss some of these methods and the theoretical background of these methods.

## 2. Materials and Methods

### 2.1. Basic Definition of Hemodynamic Parameters of Brain Tissue

The parameters of cerebral hemodynamics mainly include the following elements: CBF (cerebral blood flow), CBV (cerebral blood volume), CMRO_2_ (cerebral metabolic rate of oxygen), and OEF (oxygen extraction fraction). CBF refers to the blood flow into the vascular structure of the cerebral in the relevant area per unit of time [31]. It reflects the condition of cerebral blood flow and cerebral tissue perfusion and represents the condition of blood oxygen supply to the cerebral. It is limited by both physiological and pathological conditions of the cerebral blood supply system and is influenced by neuronal activity in the relevant brain regions. CBV is defined as the volume occupied by intravascular blood within a particular quantity of brain tissue [32]. To a certain extent, its value can reflect the expansion of blood vessels and the ability of cerebral blood flow storage. The study of Raichle et al. showed that in the resting state, the brain tissue can reflect the basic level of neuronal activity relatively stable [20]. The main parameters of brain hemodynamics meet the following equation: CMRO_2_ = OEF · CBF · Ca [33–35], where Ca represents arterial oxygen content. It is the sum of the oxygen content of red blood cells and plasma, including both oxygen bound in hemoglobin (HbO_2_) and physical dissolved oxygen. In normal state, the oxygen supply and consumption of brain tissue are in a dynamic balance, but in pathological state, such as ischemic stroke, brain trauma, or shock, the oxygen supply or consumption will be abnormal, and the balance of oxygen supply and demand will be broken; a series of changes will occur in various parameters of hemodynamics. The changing relationship between them can be shown intuitively in Figure 1.

It is assumed that when ischemic cerebrovascular disease (stroke) occurs, the CBF of the patient will be reduced to some extent, and the oxygen supply to the corresponding tissues will be reduced. And human brain tissue is a complete ability of self-adjusting system. In order to ensure the level of oxygen content required by the normal operation of human body, it will compensate by increasing the value of OEF, to maintain the CMRO_2_ at a normal level. According to the experimental studies of many scholars, the OEF of human brain is about 40% in normal condition [20], and the maximum cannot exceed 100%. Ibaraki et al. measured the OEF of healthy adults using 2D PET and found that the OEF value of gray matter under resting state was 0.35 ± 0.06 [36]. Hattori et al. measured the whole brain OEF value of healthy adults in resting state by PET as 0.39 ± 0.06 [37]. When the CBF continues to decrease, the OEF will continue to rise and reach the limit, and the brain will lose its compensation effect, resulting in the CMRO_2_ which has to decrease. At this time, the brain tissue will be in a relatively dangerous state. The decrease of CMRO_2_ indicates that the brain will face the threat of ischemic brain death, and the brain function will be abnormal due to the lack of energy supply caused by insufficient oxygen supply. If the situation of prolonged ischemia is not improved accordingly, the brain will form permanent and irreversible brain tissue damage [22]. It can be known from the brain hemodynamics that quantitative evaluation of OEF can provide insight into the pathophysiological status of many diseases. Therefore, the quantitative assessment of OEF is essential for the in-depth understanding of the disease and its subsequent treatment.

### 2.2. BOLD Effect Model

Blood oxygenation level-dependent functional magnetic resonance imaging (BOLD fMRI) technology was proposed in the 1990s, which triggered a revolution in the field of neuroimaging [38–41]. In the brain stimulated by visual and motor tasks, the possibility of using BOLD-based contrast mapping nerve activation MRI technology has been confirmed. For this reason, fMRI (functional magnetic resonance imaging) is widely considered to be the primary nondestructive measure of brain function. fMRI acquisition technology can detect signal changes, which reflect the functional changes of blood oxygen, cerebral blood flow, and cerebral blood volume. Compared with other techniques, BOLD fMRI can measure regional differences in oxygenated blood, and because of its sensitivity and spatial specificity, it has been the most widely used in functional magnetic resonance imaging.

BOLD fMRI is based on spatial segmentation of brain function. BOLD fMRI does not provide a direct way to measure neural activity; it is a local cerebral vascular oxygenation index. In BOLD imaging, deoxyhemoglobin acts as an intrinsic MRI contrast agent. MRI signal can detect the changes of deoxyhemoglobin content and functional activation. Alterations in the T2 (transverse relaxation time) or T2^∗^ (apparent transverse relaxation time) signal caused by changes in deoxyhemoglobin content form the basis of BOLD imaging.

BOLD effects can be classified as positive BOLD effects and negative BOLD effects. As neural activity increases, oxygen consumption begins to increase due to increased metabolic demand. By increasing the concentration of deoxyhemoglobin and reducing the concentration of oxyhemoglobin, this in turn changes the concentration of oxyhemoglobin and deoxyhemoglobin in the surrounding blood vessels. Deoxyhemoglobin contains four unpaired electrons and has a large magnetic moment. It is a strong paramagnetic material. It produces a magnetic gradient around and inside the blood vessel, shortens the transverse magnetization T2 or T2^∗^, and then, reduces the intensity of BOLD signal. This is the reason why an original signal change can be observed in fMRI. After the original signal changes (about 2 seconds), the enhanced neural activity will lead to a large increase in local blood flow. This increase leads to a corresponding increase in oxygen consumption. Usually, oxygen consumption is overcompensated in most parts, and excess oxygenated blood is sent to the tissues, which causes an increase in oxygenated hemoglobin. Because oxyhemoglobin is diamagnetic, and the magnetic coefficient difference between oxyhemoglobin and its surrounding tissue is very small, the local magnetic field inhomogeneity is smaller than that without neural activity. Therefore, the signal will increase and a positive BOLD effect will appear in these overcompensated areas. But if the supply of oxygen is less than the consumption, the local oxygen concentration will decrease, which in turn increases the concentration of deoxyhemoglobin in some areas. The increase in the concentration of deoxyhemoglobin will cause greater local magnetic field inhomogeneity than without neural activity. Therefore, the signal strength will be reduced at this time, and a negative BOLD effect will appear. The negative BOLD effect is the theoretical basis of MRI measurement of OEF [42].

Through sensory, motor, visual, or cognitive simulation of neural activities, the changes of magnetic resonance (MR) signal can be studied as a function of time to locate the location of the stimulation area in the brain.  Figure 2 shows the hemodynamic changes associated with brain activity [43]. Therefore, BOLD fMRI is also described as an imaging technique to characterize the specific changes of some brain diseases by analyzing the temporal and spatial characteristics of BOLD signals [44].

One of the experimental methods to quantify cerebral hemodynamic characteristics is quantitative BOLD (qBOLD). This technique was proposed by He and Yablonskiy [45]. The model is based on a multicomponent approach, including contributions from intracellular water, interstitial fluid (ISF) or cerebrospinal fluid (CSF) with resonance frequency shift, and intravascular blood. In this model, bold effects are analyzed and correlated with hemodynamic parameters such as deoxyhemoglobin concentration and OEF. It was verified on the animal model in [46] and allowed to plot hemodynamic parameters such as OEF and deoxycerebral blood volume (dCBV). In vivo studies [47–50] have also demonstrated the feasibility of this method.

## 3. MRI Scan Sequences

### 3.1. GESSE

The order of applying pulses in MRI is to give 90-degree pulses first, followed by 180-degree pulses, which is called a SE sequence (spin-echo sequence). Conventional SE sequence have high signal-to-noise ratio (SNR) T2 signals, but these signals are not sensitive to the magnetic susceptibility changes caused by oxygen metabolism in brain tissues. GRE sequence (gradient recalled echo sequence) is a pulse sequence that generates an echo signal and generates an image using a switch in the direction of the gradient field after RF (radio frequency) excitation. Its RF excitation angle is generally less than 90° to obtain a large transverse magnetization vector in a short longitudinal recovery time. However, due to the rapid change of direction of gradient magnetic field during the signal acquisition in the conventional GRE sequence, hydrogen proton phase loss rate is faster than that in the SE sequence, the obtained echo signal is actually T2^∗^ signal, and the oxygen metabolism factor of brain tissue that needs to be extracted is mixed with other factors, which is also not obvious. Therefore, it is necessary to have a scanning sequence that simultaneously obtains T2 and T2^∗^ signals to extract the difference in magnetic susceptibility caused by oxygen metabolism of brain tissue, reflect the quantity changes of the two kinds of hemoglobin, and display the functional metabolism information of brain activity clearly and accurately. Based on this consideration, the traditional SE and GRE sequences cannot extract the T2 and T2^∗^ signals at the same time. Therefore, part of the pulses in SE and GRE sequences are modified and recombined, namely, the GESSE sequence. T2 and T2^∗^ signals can be obtained simultaneously by one sequence, which is convenient to separate T2′ from the model.

GESSE (gradient echo sampling of spin echo) sequence is based on the traditional SE sequence, which changes the original single echo acquisition spin echo center to use multiple unipolar gradients to quickly switch sampling the whole spin echo process. The idea of this sequence was first published by Yablonskiy and Haacke [51]. They improved the GESFIDE (gradient echo sampling of FID and echo) sequence of Ma and Wehrli [52] and changed the acquisition of FID (free induction decay) signal to acquisition of echo signal only. The reason for this is that in general, due to the refocusing effect of 180-degree radio frequency pulse, there is a specific symmetrical MR signal on both sides of the spin echo, which is not sensitive to the inhomogeneity of the magnetic field and is more accurate for T2 measurement. The signal is usually collected at the center of the echo. At this time, the T2 signal is obtained without the influence of the difference in magnetic susceptibility [53]. When a series of gradient echo samples are used on both sides of the spin echo center, all the echo signals except the spin echo position are T2^∗^ signals containing local magnetic susceptibility difference. So, T2 and T2^∗^ signals can be obtained at the same time. The sequence diagram is shown in Figure 3.

The GESSE sequence is based on the conventional SE sequence, but with some differences, mainly in the *k*-space and readout gradient. In the *K*-space filling, the method of collecting gradients in each TR (time of repetition) is used to fill multiple *K*-spaces at the same time. In order to ensure that the postprocessing data contains enough signals, the number of echoes in the echo chain is about 32. In addition, an asymmetric design can be adopted, that is, the echo number on both sides of the spin echo is not necessarily equal [45]. Under the premise of ensuring the echo number of the shortest time scale, the spin echo is moved forward as far as possible, in order to collect the signal when the signal intensity is high and improve the signal-to-noise ratio of the image. A readout gradient in the sequence corresponds to a row in the *k*-space frequency coding direction. The GESSE sequence uses 32 gradients (corresponding to 32 images), so the GESSE sequence fills the same row in 32 *k*-spaces simultaneously in one TR, as shown in Figure 4.

In the data collection part, it can be seen from the sequence diagram that the collection method is similar to that of SE-EPI (spin-echo echo planar imaging). However, it should be noted that GESSE sequence does not collect echoes at every positive and negative gradient. Due to the inevitable influence of system instability, if a rapid switch is made from a positive gradient to a negative gradient, the phase shift of the magnetization vector in the *X*-*Y* plane will exist compared with the phase shift in the positive gradient [54]. At this time, we get the image as shown in Figure 5. There will be position difference between the odd and even images after reconstruction in the phase coding direction, which is similar to the common N/2 artifacts in EPI (echo planar imaging) acquisition.

In order to solve the problem of phase error, the method of unipolar gradient collection is adopted, that is, the collection is only performed when the gradient is positive or negative. For example, only the positive gradient is used as the readout gradient of the acquired image, and a negative gradient equal to its area is added between each positive readout gradient as the wraparound gradient. In this way, a series of images without phase shift can be obtained, as shown in Figure 6.

GESSE has been used to assess the misery perfusion of patients with cerebral ischemia and obtain reliable brain OEF results [55]. Lei et al. applied this promising method to study the brain OEF of MELAS patients at different stages and confirmed that MRI can quantitatively show the changes in OEF at different stages of stroke-like episodes [56]. Meng et al. scanned the normal human brains of different ages with GESSE sequence and measured OEF value, which confirmed that GESSE sequence can accurately measure OEF value of human brain. There was no significant difference in OEF value between gray matter and white matter of normal human brain; only gray matter OEF value increased slightly with age [57]. Domsch et al. used GESSE sequence to collect in vivo data from five healthy volunteers and one patient with primary brain tumor at 3 T and used simulated BOLD data to train the ANN. Achieve OEF mapping with reduced variance, which helps to integrate it into clinical protocols [58].

GESSE sequence still has the following shortcomings: (1) the scanning time is long and motion artifacts are easy to appear; (2) it can only be scanned by single layer, and the scanning range is limited; (3) it is easy to be affected by the inhomogeneity of magnetic field; (4) the hematocrit value is set as a fixed value, but in practice, due to individual differences and different physiological conditions, the final measurement error may occur.

### 3.2. MEGESE

In 2000, An and Lin used MEGESE (multiecho gradient echo/spin echo) sequence to simultaneously measure the values of T2 and T2^∗^ in a TR interval and, based on this, calculated brain OEF by using two-compartment model [59]. The sequence consists of 21 echoes, all of which are obtained after the *π* pulse, the eleventh echo is a spin echo (SE), and all the other echoes are gradient echo (GE) and are placed symmetrically on both sides of the SE. The MEGESE sequence diagram is shown in Figure 7 [59].

An et al. used 2D MEGESE sequence to prove that quantitative cerebral blood oxygen saturation (CBOS) can be obtained by MRI, and the CBOS measured by MRI can be converted into brain OEF, which is very consistent with the results reported in PET literature [60, 61]. Lee et al. used the 2D MEGESE sequence to obtain a slice in the center of the lesion based on the DWI (diffusion-weighted imaging) at tp1 (4.5 ± 0.9 hours), tp2 (3 to 5 days), and tp3 (1 to 3 months), which was then used to obtain the estimated value of OEF [62]. This method has good consistency between the OEF measurement results of normal people and the PET measurement results. However, this method also has many factors that limit its clinical application, such as the limited coverage of single-slice scans, long data acquisition time, and sensitive to motion artifacts. Therefore, this method has not been widely used in clinical practice.

### 3.3. ASE EPI

ASE-OEF uses an ASE EPI (single-shot asymmetric spin-echo echo-planar imaging) sequence as a fast OEF measurement sequence [63]. The ASE EPI sequence is developed on the basis of the single-shot spin-echo echo-planar imaging sequence. In the SE EPI (spin echo EPI) sequence, TE is defined as the time interval between the 90-degree pulse and the *K*-space centroid acquisition. In the ASE EPI sequence, under the condition that the TE (time of echo) remains unchanged, the 180-degree pulse shifted a *τ* time along the time axis, and the difference in time of *τ* is used to reflect the signal change caused by the magnetic sensitivity. In the ASE EPI sequence, the MR signal is not only related to the frequency shift caused by the microscopic magnetic sensitivity change caused by deoxyhemoglobin but also related to the T1 (longitudinal relaxation time) and T2. The effect of T2 on the signal can be effectively eliminated by fixing the TE time, and the effect of T1 on the signal can be eliminated by making the TR much larger than TE/2*τ*, so that the MRI signal mainly reflects the change of deoxyhemoglobin content. The ASE-EPI sequence diagram is shown in Figure 8 [63].

Chang et al. used the ASE EPI sequence to measure the changes in OEF values before and after controllable hypercapnia in dogs and proved that the sequence is reliable [64]. Subsequently, the ASE EPI sequence was used to measure the changes of OEF value of brain tissue before and after modeling of canine cerebral ischemia model, and it was verified that the sequence can successfully reflect the oxygen metabolism state of ischemic brain tissue, which will be of great significance for the evaluation of cerebral hemodynamic state of patients with cerebrovascular disease [65]. Liang et al. verified that ASE EPI sequence can be used for noninvasive measurement of OEF in tumor tissue, and quantitative index OEF can well identify high-grade and low-grade gliomas and reflect the proliferative activity of tumor to a certain extent [66]. Cui combined ASE EPI sequence with pCASL (pseudocontinuous arterial spin labeling) sequence to scan normal people and patients with acute cerebral infarction of different ages, which can initially realize one-stop assessment of human brain OEF and CBF values [67]. This method is noninvasive to the body, and the examination time is short.

Compared with MEGESE sequence, the main advantages of ASE EPI sequence are as follows: (1) the acquisition of echo number is no longer limited by TE, and the readout bandwidth is the same as MEGESE sequence; (2) because the TE time is fixed, R2 (1/T2) cannot be measured before evaluating OEF, so the measurement error associated with T2 can be avoided; (3) a single excitation of EPI reduces the artifact caused by motion; (4) EPI sequence combined with the application of flow dephasing gradient reduces the influence of intravascular signals, but does not increase the sensitivity of the gradient to motion.

Compared with GESSE sequence, ASE EPI sequence has the following advantages: (1) ASE sequence can be scanned by multiple layers; (2) the obtained echo number is no longer limited by TE and readout bandwidth; (3) TE is constant, T2 effect is constant, and R2 is constant, which reduces the error when calculating OEF; (4) the single excitation EPI method reduces the artifact caused by motion; (5) EPI method uses the flow dephasing gradient to minimize the signal contribution in blood vessels.

On the other hand, the disadvantages of this method are as follows: (1) the readout gradient of EPI is prone to high-frequency signal noise; (2) the hypothesis of random distribution of blood vessel direction may be disturbed by the presence of leptomeningeal vessels in the adjacent cortical sulcus; (3) because of the use of the two compartment model, that is to say, the extravascular brain tissue is considered to be homogeneous, the effect of cerebrospinal fluid is ignored when the cortical measurement is specially designed, thus affecting the measurement accuracy. The inaccuracy and nonquantification of the measurement limit its application.

### 3.4. TRUST

Lu and Ge et al. used TRUST (T2 relaxation under spin tagging) technology to separate pure blood signals [68]. In this method, vein end spin labeling technology similar to conventional artery spin labeling and pair subtraction processing were used, and the subtraction images obtained only included venous blood signals. The T2 of the signal is determined and converted into venous oxygenation (Yv) using the calibration curve. To reduce the quantitative assessment of the blood T2 outflow effect, the T2-weighted image uses a series of nonplanar selective T2 prepulses instead of a conventional spin echo sequence, as shown in Figure 9 [68].

The TRUST technology pulse sequence includes interlaced marks and control scan signals. Each image type requires four different effective TE times, which range from 0 to 160 ms. For each scan, the presaturated radio frequency pulse is used at the beginning of the sequence to suppress the signal from the static tissue, and then, the radio frequency pulse is marked (or controlled) to mark the incoming blood. A definite waiting time (1.2 s) is required for the blood flow imaging layer. Before data acquisition, in order to reduce the quantitative evaluation of blood T2 outflow effect, T2-weighted images used a series of nonplanar selected T2 prepulses instead of conventional spin echo sequences. The yellow region and the green region, respectively, represent the positioning of the imaging layer and the label layer using the principle of spin labeling. The signals from static tissues can be subtracted and eliminated, so the separation of pure blood signals can be achieved. Different from previous experiments, the spatial resolution of this technique is not limited by the need of vessel diameter or voxel to fit the diameter of inner cerebral veins. Therefore, the technique can minimize the partial volume effect and avoid the need of the specific selection of voxel including blood and has a better signal-to-noise ratio. However, this technique still has shortcomings. The information of this method mainly comes from the superior sagittal sinus. Due to the low blood signal intensity, the measurement of venules will show a large evaluation error. Therefore, the use of this technology to measure local Yv of the lesion needs to be further deepened.

Due to the limitation that TRUST sequences require a long repetition time, Xu et al. proposed that postsaturation T2 could relax the subspin markers by putting a nonselective 90° pulse after signal acquisition to reset the magnetization of the whole brain, thus improving the speed and reliability of TRUST technique in measuring brain oxygenation [69]. Xu et al. used TRUST technology and ASL (arterial spin labeling) technology to test the change of CBF, CMRO2, and OEF with time in 10 healthy young people aged 22-35 years after consuming 200 mg caffeine and found that CBF decreased and OEF significantly increased, while CMRO2 had no significant change [70]. Liu et al. successfully used TRUST sequence to measure Yv in multiple locations with multiple 3 T scanners, and the results showed that the sequence could be implemented and performed accurately and reliably, indicating that the technology is stable and feasible, which is a key step towards the availability and potential clinical application of cerebral oxygen metabolism measurement [71]. O'Brien et al. proposed selective localized TRUST (SL-TRUST) by adjusting the original TRUST sequence, so that the spatially specific measurement of venous blood T2 can be achieved to quantify the OEF in different regions of the brain. This method realizes the spatial positioning of the OEF in brain tissue, while still retaining the acquisition in the sagittal sinus [72]. Jiang et al. compared the values measured by TRUST and gold standard ^15^O-PET to evaluate the accuracy of whole brain OEF estimation based on T2. The whole brain OEF measured by TRUST is very consistent with that measured by gold standard ^15^O-PET, with high accuracy and repeatability, which proves that TRUST MRI can accurately quantify whole brain OEF noninvasively [73].

The advantage of TRUST technology is that the measurement results are less affected by other tissues, because the images generated by static tissues can be removed by subtracting the control image and the label image in the later data processing. Thus, TRUST results are displayed independent of imaging resolution [66], and independent of the range of the region of interest manually selected by the operator. A good agreement between Yv values measured by TRUST and those measured by other techniques has been reported in the literature [74–76]. The results of Yv measured by trust sequence have no significant change on head motion and blood signal intensity compared with other MRI sequences. Therefore, using TRUST sequence to measure human brain OEF is less demanding than other sequences. At the same time, the scanning time of the TRUST sequence is relatively short (about 1.2 min). These features allow the TRUST technique to be widely used for noninvasive detection of brain activity since the measurement of whole brain OEF. It should be noted, however, that the technique still has drawbacks, as the method information is mainly derived from the superior sagittal sinus, and the measurement of small veins will exhibit a large assessment error due to the lower blood signal intensity. Therefore, the measurement of the local Yv of the lesion using this technique needs to be further deepened.

### 3.5. QUIXOTIC

Bolar et al. proposed a QUantitative Imaging of eXtraction of oxygen and TIssue consumption (QUIXOTIC) to measure OEF [77]. The method used velocity-selective spin labeling (VSSL) to isolate blood signals from the posterior capillary venules (PCV). In principle, the method uses velocity-sensitive pulses to collect the nonuniform flow velocity and single-phase flow in the venous tree, thus establishing the blood flow dependent on venous blood components. This sequence uses a T2-based preparation technique to obtain PCV blood weighted images at effective echo time and perform exponential fitting on these data to estimate T2 of PCV blood. The function relationship between T2 value and blood oxygen saturation was established to calculate OEF. The method could also measure CBF at the same time and calculate CMRO2 accordingly. The sequence diagram is shown in Figure 10.

Since QUIXOTIC measures the OEF in the voxel direction with a long scanning time, which limits its application, Stout et al. proposed a multiecho QUIXOTIC called turbo QUIXOTIC (tQUIXOTIC), which reduces the scanning time by eight times and applies it to functional MRI [78]. This method can obtain multiple echo readings in a single TR, thereby shortening the imaging time by several times, so that the cortical GM OEF mapping can be completed in 3.4 minutes, and the OEF time course of functional MRI is generated.

The advantages of QUIXOTIC include the following: (1) QUIXOTIC only maps blood in the venous circulation, eliminating interference such as cerebrospinal fluid, static tissue, and capillary/arterial blood; (2) due to the limitation of signal-to-noise ratio, QUIXOTIC analysis can be performed on a voxel-per-voxel basis to create Yv, OEF, and CMRO_2_ mapping; (3) QUIXOTIC generates images every two TR, thus enabling the technology to be used in functional MRI.

Based on the several sequences discussed above, their advantages and disadvantages are summarized as shown in Table 1.

## 4. Discussion

This paper discusses the progress of MRI studies of OEF in human brain. However, due to the internal small signal changes caused by deoxyhemoglobin and the influence of various confounding factors, these techniques need to be further improved as routine clinical diagnostic tools. In addition, a series of physiological and pathological conditions are required to strictly compare and verify the technology. In today's fast-developing era, various technical methods cannot be described in detail due to limited knowledge and experience, so we can only briefly describe the new methods which are widely used in recent years. It is hoped that this review can provide relevant background knowledge for relevant researchers and medical staff, to select an appropriate method for relevant medical experiments and provide a new way for clinical diagnosis and treatment. Meanwhile, we hope it will promote the innovation and development of in vivo quantitative nuclear magnetic resonance technology for measuring human brain OEF in the future.

## 5. Conclusion

Cerebral oxygen metabolism plays an important role in maintaining normal brain function and is the basic energy source for maintaining neural function. Because the brain has very limited energy stores, a relatively short period of disturbance in cerebral oxygen metabolism may cause serious damage to tissue, such as a stroke. Quantitative measurement of tissue oxygenation and oxygen metabolism is very important for understanding the pathophysiological status and treatment of many diseases. As one of the important parameters of hemodynamic and tissue metabolic conditions of human brain, OEF can indirectly reflect the physiological condition of brain tissue and the degree of lesions and can be used as an auxiliary criterion of disease in clinical diagnosis. Therefore, this review summarizes some principles and methods of MRI for quantitative measurement of OEF based on the BOLD principle and discusses the advantages and disadvantages of each method. It is suggested that follow-up scholars can improve the OEF measurement technology and methods based on MRI according to the discussion in this paper.

## Figures and Tables

**Figure 1:** The relationship between the parameters of cerebral hemodynamics.

**Figure 2:** Hemodynamic changes in brain activity [43].

**Figure 3:** GESSE sequence timing diagram.

**Figure 4:** GESSE sequence *K* space filling method.

**Figure 5:** The image with phase error acquired by using positive and negative gradient echo.

**Figure 6:** Phase error-free images acquired with unipolar gradient acquisition.

**Figure 7:** MEGESE sequence diagram.

**Figure 8:** ASE-EPI sequence diagram.

**Figure 9:** Schematic diagram of TRUST technology pulse sequence.

**Figure 10:** QUIXOTIC sequence diagram.

**Table 1:** Summary of MRI scan sequences.

Sequence	Advantages	Disadvantages
GEESE (gradient-echo sampling of spin echo)	Scan sequences of T2 and T2^∗^ signals can be obtained simultaneously as a way to extract differences in magnetization rates resulting from oxygen metabolism in brain tissue, reflect changes in the amounts of the two types of hemoglobin, and display functional metabolic information about brain activity in a clear and accurate manner.	(1) The scanning time is long and motion artifacts are easy to appear; (2) it can only be scanned by single layer, and the scanning range is limited; (3) it is easy to be affected by the inhomogeneity of magnetic field; (4) the hematocrit value is set as a fixed value, but in practice, due to individual differences and different physiological conditions, the final measurement error may occur

MEGESE (multiecho gradient echo/spin echo)	This method has good consistency between the OEF measurement results of normal people and the PET measurement results.	(1) Limited coverage of single-slice scans; (2) long data acquisition time; (3) sensitive to motion artifacts.

ASE-EPI (single-shot asymmetric spin-echo echo-planar imaging)	(1) ASE sequence can be scanned by multiple layers; (2) the obtained echo number is no longer limited by TE and readout bandwidth; (3) TE is constant, T2 effect is constant, R2 is constant, which reduces the error when calculating OEF; (4) the single excitation EPI method reduces the artifact caused by motion; (5) EPI method uses the flow dephasing gradient to minimize the signal contribution in blood vessels	(1) The readout gradient of EPI is prone to high-frequency signal noise; (2) the hypothesis of random distribution of blood vessel direction may be disturbed by the presence of leptomeningeal vessels in the adjacent cortical sulcus; (3) because of the use of the two compartment model, that is to say, the extravascular brain tissue is considered to be homogeneous, the effect of cerebrospinal fluid is ignored when the cortical measurement is specially designed, thus affecting the measurement accuracy

TRUST (T2 relaxation under spin tagging)	The measurement results are less affected by other tissues, because the images generated by static tissues can be removed by subtracting the control image and the label image in the later data processing. Thus, TRUST results are displayed independent of imaging resolution and independent of the range of the region of interest manually selected by the operator.	The method information is mainly derived from the superior sagittal sinus, and the measurement of small veins will exhibit a large assessment error due to the lower blood signal intensity. Therefore, the measurement of the local Yv of the lesion using this technique needs to be further deepened.

QUIXOTIC (quantitative imaging of extraction of oxygen and tissue consumption)	(1) QUIXOTIC only maps blood in the venous circulation, eliminating interference such as cerebrospinal fluid, static tissue and capillary/arterial blood; (2) due to the limitation of signal-to-noise ratio, QUIXOTIC analysis can be performed on a voxel-per-voxel basis to create Yv, OEF, and CMRO2 mapping; (3) QUIXOTIC generates images every two TR, thus enabling the technology to be used in functional MRI	It has a long scan duration—only one TE (time of echo) is acquired for each TR (time of repetition). And it requires several repetitions to obtain sufficient SNR to determine T2 over the required number of TEs. And the OEF values converted from Yv differences are lower than those measured by TRUST due to bias from the QUIXOTIC technique itself and the inevitable diffusion weighting in the experiment.

## Data Availability

The data used to support the findings of this study are included within the article.

## References

[1] Feng X., Ge Y., Lu H. (2009). Noninvasive quantification of whole-brain cerebral metabolic rate of oxygen (CMRO2) by MRI. *Magnetic Resonance in Medicine*.

[2] Sheng X. (2014). MR OEF imaging in MELAS. *Methods in Enzymology*.

[3] Raichle M. E., Gusnard D. A. (2002). Appraising the brain's energy budget. *Proceedings of the National Academy of Sciences of the United States of America*.

[4] Cho J., Zhang S., Kee Y. (2020). Cluster analysis of time evolution (CAT) for quantitative susceptibility mapping (QSM) and quantitative blood oxygen level-dependent magnitude (qBOLD)-based oxygen extraction fraction (OEF) and cerebral metabolic rate of oxygen (CMRO2) mapping. *Magnetic Resonance in Medicine*.

[5] Stadlbauer A., Zimmermann M., Kitzwögerer M. (2017). MR imaging-derived oxygen metabolism and neovascularization characterization for grading and *IDH* gene mutation detection of gliomas. *Radiology*.

[6] Preibisch C., Shi K., Kluge A. (2017). Characterizing hypoxia in human glioma: a simultaneous multimodal MRI and PET study. *NMR in Biomedicine*.

[7] Wiestler B., Kluge A., Lukas M. (2016). Multiparametric MRI-based differentiation of WHO grade II/III glioma and WHO grade IV glioblastoma. *Scientific Reports*.

[8] Derdeyn C. P., Videen T. O., Yundt K. D. (2002). Variability of cerebral blood volume and oxygen extraction: stages of cerebral haemodynamic impairment revisited. *Brain*.

[9] An H., Ford A. L., Vo K. D. (2014). Imaging oxygen metabolism in acute stroke using MRI. *Current Radiology Reports*.

[10] Ibaraki M., Shimosegawa E., Miura S. (2004). PET measurements of CBF, OEF, and CMRO2 without arterial sampling in hyperacute ischemic stroke: method and error analysis. *Annals of Nuclear Medicine*.

[11] Iadecola C. (2004). Neurovascular regulation in the normal brain and in Alzheimer's disease. *Nature Reviews Neuroscience*.

[12] Iadecola C. (2005). Rescuing troubled vessels in Alzheimer disease. *Natural Medicine*.

[13] Vlassenko A. G., Vaishnavi S. N., Couture L. (2010). Spatial correlation between brain aerobic glycolysis and amyloid-*β* (A*β*) deposition. *Proceedings of the National Academy of Sciences of the United States of America*.

[14] Powers W. J., Videen T. O., Markham J. (2007). Selective defect of in vivo glycolysis in early Huntington's disease striatum. *Proceedings of the National Academy of Sciences of the United States of America*.

[15] Beal M. F. (1998). Mitochondrial dysfunction in neurodegenerative diseases. *Biochimica et Biophysica Acta*.

[16] Leenders K. L., Frackowiak R. S., Quinn N., Marsden C. D. (1986). Brain energy metabolism and dopaminergic function in Huntington's disease measured in vivo using positron emission tomography. *Movement Disorders*.

[17] Santens P., De Reuck J., Crevits L. (2004). Cerebral oxygen metabolism in patients with progressive supranuclear palsy: a positron emission tomography study. *European Neurology*.

[18] Shishido F., Uemura K., Inugami A. (1996). Cerebral oxygen and glucose metabolism and blood flow in mitochondrial encephalomyopathy: a PET study. *Neuroradiology*.

[19] Tanaka M., Kondo S., Okamoto K., Hirai S. (1997). Cerebral perfusion and oxygen metabolism in Parkinson's disease: positron emission tomographic study using oxygen-15-labeled CO2 and O2. *Nihon Rinsho Japanese Journal of Clinical Medicine*.

[20] Raichle M. E., MacLeod A. M., Snyder A. Z., Powers W. J., Gusnard D. A., Shulman G. L. (2001). A default mode of brain function. *Proceedings of the National Academy of Sciences*.

[21] Gusnard D. A., Raichle M. E., Raichle M. E. (2001). Searching for a baseline: functional imaging and the resting human brain. *Nature Reviews Neuroscience*.

[22] Powers W. J., Grubb R. L., Raichle M. E. (1984). Physiological responses to focal cerebral ischemia in humans. *Annals of Neurology*.

[23] Yablonskiy D. A., Sukstanskii A. L., He X. (2013). Blood oxygenation level-dependent (BOLD)-based techniques for the quantification of brain hemodynamic and metabolic properties – theoretical models and experimental approaches. *NMR in Biomedicine*.

[24] Mintun M. A., Raichle M. E., Martin W. R., Herscovitch P. (1984). Brain oxygen utilization measured with O-15 radiotracers and positron emission tomography. *Journal of Nuclear Medicine*.

[25] Altman D. I., Lich L. L., Powers W. J. (1991). Brief inhalation method to measure cerebral oxygen extraction fraction with PET: accuracy determination under pathologic conditions. *Journal of Nuclear Medicine*.

[26] Ishii K., Kitagaki H., Kono M., Mori E. (1996). Decreased medial temporal oxygen metabolism in Alzheimer’s disease shown by PET. *Journal of Nuclear Medicine*.

[27] Wintermark M., Sesay M., Barbier E. (2005). Comparative overview of brain perfusion imaging techniques. *Stroke*.

[28] Herscovitch P., Markham J., Raichle M. E. (1983). Brain blood flow measured with intravenous H2(15)O. I. Theory and error analysis. *Journal of Nuclear Medicine*.

[29] Matsubara K., Ibaraki M., Shinohara Y., Takahashi N., Toyoshima H., Kinoshita T. (2021). Prediction of an oxygen extraction fraction map by convolutional neural network: validation of input data among MR and PET images. *International Journal of Computer Assisted Radiology and Surgery*.

[30] Wang X., Sukstanskii A. L., Yablonskiy D. A. (2013). Optimization strategies for evaluation of brain hemodynamic parameters with qBOLD technique. *Magnetic Resonance in Medicine*.

[31] Zazulia A. R., Markham J., Powers W. J. (2004). Cerebral blood flow and metabolism in human cerebrovascular disease. *Stroke: Pathophysiology, diagnosis, and management*.

[32] Vagal A., Vossough A., Lev M. H., Wintermark M. (2016). *Handbook of Neuro-Oncology Neuroimaging (Second Edition)*.

[33] Attwell D., Laughlin S. B. (2001). An energy budget for signaling in the grey matter of the brain. *Journal of Cerebral Blood Flow and Metabolism*.

[34] Kety S. S., Schmidt C. F. (1948). The nitrous oxide method for the quantitative determination of cerebral blood flow in man: theory, procedure and normal values 1. *The Journal of Clinical Investigation*.

[35] Powers W. J., Grubb R. L., Darriet D., Raichle M. E. (1985). Cerebral blood flow and cerebral metabolic rate of oxygen requirements for cerebral function and viability in humans. *Journal of Cerebral Blood Flow and Metabolism*.

[36] Ibaraki M., Miura S., Shimosegawa E. (2008). Quantification of cerebral blood flow and oxygen metabolism with 3-dimensional PET and 15O: validation by comparison with 2-dimensional PET. *Journal of Nuclear Medicine*.

[37] Hattori N., Bergsneider M., Wu H. M. (2004). Accuracy of a method using short inhalation of (15)O-O(2) for measuring cerebral oxygen extraction fraction with PET in healthy humans. *Journal of Nuclear Medicine*.

[38] Thulborn K. R., Waterton J. C., Matthews P. M., Radda G. K. (1982). Oxygenation dependence of the transverse relaxation time of water protons in whole blood at high field. *Biochimica et Biophysica Acta*.

[39] Ogawa S., Lee T. M., Tank A. (1990). Brain magnetic resonance imaging with contrast dependent on blood oxygenation. *Proceedings of the National Academy of Sciences of the United States of America*.

[40] Ogawa S., Lee T. M., Barrere B. (1993). The sensitivity of magnetic resonance image signals of a rat brain to changes in the cerebral venous blood oxygenation. *Magnetic Resonance in Medicine*.

[41] Ogawa S., Menon R. S., Tank D. W. (1993). Functional brain mapping by blood oxygenation level-dependent contrast magnetic resonance imaging. A comparison of signal characteristics with a biophysical model. *Biophysical Journal*.

[42] Nair D. G. (2005). About being BOLD. *Brain Research Reviews*.

[43] He L. (2008). *MRI/FMRI Noise Reduction and Data Analysis*.

[44] Fox M. D., Raichle M. E. (2007). Spontaneous fluctuations in brain activity observed with functional magnetic resonance imaging. *Nature Reviews Neuroscience*.

[45] He X., Yablonskiy D. A. (2007). Quantitative BOLD: mapping of human cerebral deoxygenated blood volume and oxygen extraction fraction: default state. *Magnetic Resonance in Medicine*.

[46] He X., Zhu M., Yablonskiy D. A. (2008). Validation of oxygen extraction fraction measurement by qBOLD technique. *Magnetic Resonance in Medicine*.

[47] Dickson J. D., Ash T., Williams G. B. (2010). Quantitative BOLD: the effect of diffusion. *Journal of Magnetic Resonance Imaging*.

[48] Sedlacik J., Reichenbach J. R. (2010). Validation of quantitative estimation of tissue oxygen extraction fraction and deoxygenated blood volume fraction in phantom and in vivo experiments by using MRI. *Magnetic Resonance in Medicine*.

[49] Sohlin M. C., Schad L. R. (2011). Susceptibility-related MR signal dephasing under nonstatic conditions: experimental verification and consequences for qBOLD measurements. *Journal of Magnetic Resonance Imaging*.

[50] Cho J., Lee J., An H., Goyal M. S., Su Y., Wang Y. (2021). Cerebral oxygen extraction fraction (OEF): comparison of challenge-free gradient echo QSM+qBOLD (QQ) with 15O PET in healthy adults. *Journal of Cerebral Blood Flow and Metabolism*.

[51] Yablonskiy D. A., Haacke E. M. (1997). An MRI method for measuring T2 in the presence of static and RF magnetic field inhomogeneities. *Magnetic Resonance in Medicine*.

[52] Ma J. F., Wehrli F. W. (1996). Method for image-based measurement of the reversible and irreversible contribution to the transverse-relaxation rate. *Journal of Magnetic Resonance Series B*.

[53] Yablonskiy D. A., Haacke E. M. (1994). Theory of NMR signal behavior in magnetically inhomogeneous tissues: the static dephasing regime. *Magnetic Resonance in Medicine*.

[54] Yablonskiy D. A. (1998). Quantitation of intrinsic magnetic susceptibility-related effects in a tissue matrix. Phantom study. *Magnetic Resonance in Medicine*.

[55] Xie S., Hui L. H., Xiao J. X., Zhang X. D., Peng Q. (2011). Detecting misery perfusion in unilateral steno-occlusive disease of the internal carotid artery or middle cerebral artery by MR imaging. *American Journal of Neuroradiology*.

[56] Yu L., Xie S., Xiao J., Wang Z., Zhang X. (2013). Quantitative measurement of cerebral oxygen extraction fraction using MRI in patients with MELAS. *PLoS One*.

[57] Meng L. L., Zou Y., Zhang X. D. (2011). MRI measurement of brain oxygen extraction fraction in normal subjects. *Chinese Journal of Medical Imaging Technology*.

[58] Domsch S., Mürle B., Weingärtner S., Zapp J., Wenz F., Schad L. R. (2018). Oxygen extraction fraction mapping at 3 tesla using an artificial neural network: a feasibility study. *Magnetic Resonance in Medicine*.

[59] An H., Lin W. (2000). Quantitative measurements of cerebral blood oxygen saturation using magnetic resonance imaging. *Journal of Cerebral Blood Flow and Metabolism*.

[60] An H., Lin W. (2002). Cerebral oxygen extraction fraction and cerebral venous blood volume measurements using MRI: effects of magnetic field variation. *Magnetic Resonance in Medicine*.

[61] An H., Lin W., Celik A., Lee Y. Z. (2001). Quantitative measurements of cerebral metabolic rate of oxygen utilization using MRI: a volunteer study. *NMR in Biomedicine*.

[62] Lee J. M., Vo K. D., An H. (2003). Magnetic resonance cerebral metabolic rate of oxygen utilization in hyperacute stroke patients. *Annals of Neurology*.

[63] An H., Lin W. (2003). Impact of intravascular signal on quantitative measures of cerebral oxygen extraction and blood volume under normo- and hypercapnic conditions using an asymmetric spin echo approach. *Magnetic Resonance in Medicine*.

[64] Chang F., Xie S., Zhang Z. (2016). ASE in measuring oxygen extraction fraction change in canine brain under hypercapnia. *Chinese Journal of Medical Imaging Technology*.

[65] Chang F., Xie S., Yu L., Cheng S., Zhang Z., Wang W. (2016). Quantitative measurement of cerebral oxygen metabolism using asymmetric spin echo version of echo planar imaging sequence in an animal model of ischemia. *Chinese Journal of Radiology*.

[66] Liang S. C., Zhang J. X., Zhang S. (2016). The application of MR oxygen extraction fraction imaging in astrocytoma grading. *Chinese Journal of Magnetic Resonance Imaging*.

[67] Cui L. Y. (2015). *The MRI Study of Brain Oxygen Extraction Fraction and Cerebral Blood Flow in Normal Subjects and Patients with Acute Cerebral Infarction*.

[68] Lu H., Ge Y. (2008). Quantitative evaluation of oxygenation in venous vessels using T2-relaxation- under-spin-tagging MRI. *Magnetic Resonance in Medicine*.

[69] Xu F., Uh J., Liu P., Lu H. (2012). On improving the speed and reliability of T2-relaxation-under-spin-tagging (TRUST) MRI. *Magnetic Resonance in Medicine*.

[70] Xu F., Liu P., Pekar J. J., Lu H. (2015). Does acute caffeine ingestion alter brain metabolism in young adults?. *NeuroImage*.

[71] Liu P., Dimitrov I., Andrews T. (2016). Multisite evaluations of a T2-relaxation-under-spin-tagging (TRUST) MRI technique to measure brain oxygenation. *Magnetic Resonance in Medicine*.

[72] O'Brien C., Okell T. W., Chiew M., Jezzard P. (2019). Volume-localized measurement of oxygen extraction fraction in the brain using MRI. *Magnetic Resonance in Medicine*.

[73] Jiang D., Deng S., Franklin C. G. (2021). Validation of T2-based oxygen extraction fraction measurement with 15O positron emission tomography. *Magnetic Resonance in Medicine*.

[74] Jain V., Langham M. C., Wehrli F. W. (2010). MRI estimation of global brain oxygen consumption rate. *Journal of Cerebral Blood Flow and Metabolism*.

[75] Qin Q., Grgac K., van Zijl P. C. (2011). Determination of whole-brain oxygen extraction fractions by fast measurement of blood T2 in the jugular vein. *Magnetic Resonance in Medicine*.

[76] Ito H., Kanno I., Kato C. (2004). Database of normal human cerebral blood flow, cerebral blood volume, cerebral oxygen extraction fraction and cerebral metabolic rate of oxygen measured by positron emission tomography with 15O-labelled carbon dioxide or water, carbon monoxide and oxygen: a multicentre study in Japan. *European Journal of Nuclear Medicine and Molecular Imaging*.

[77] Bolar D. S., Rosen B. R., Sorensen A. G., Adalsteinsson E. (2011). QUantitative Imaging of eXtraction of oxygen and TIssue consumption (QUIXOTIC) using venular-targeted velocity-selective spin labeling. *Magnetic Resonance in Medicine*.

[78] Stout J. N., Adalsteinsson E., Rosen B. R., Bolar D. S. (2017). Functional oxygen extraction fraction (OEF) imaging with turbo gradient spin echo QUIXOTIC (turbo QUIXOTIC). *Magnetic Resonance in Medicine*.

